# Wavelet Transform-Based Ultrasound Image Enhancement Algorithm for Guided Gynecological Laparoscopy Imaging of Local Anesthetics in Perioperative Gynecological Laparoscopy

**DOI:** 10.1155/2021/5169803

**Published:** 2021-07-22

**Authors:** Bingbing Sheng, Qiaoqin Yan, Xianda Zhao, Wujian Yang

**Affiliations:** Department of Anaesthesiology, The First People's Hospital of Wenling, Taizhou 317500, Zhejiang, China

## Abstract

This paper aimed to study the application of local anesthetics combined with transversus abdominis plane (TAP) block in gynecological laparoscopy (GLS) surgery during perioperative period under the guidance of ultrasound image enhanced by the wavelet transform image enhancement (WTIE) algorithm. 56 patients who underwent GLS surgery in hospital were selected and classified as the infiltrating group and block group. The puncture needle was guided by ultrasound images under WTIE algorithm, and 0.375% ropivacaine was adopted to block TAP. The results showed that the dosage of propofol in the infiltrating group (313.23 ± 19.67 mg) was remarkably inferior to the infiltrating group (377.67 ± 21.56 mg) (*P* < 0.05). The hospitalization time of patients in the infiltrating group (2.14 ± 0.18 days) was obviously shorter than that of the infiltrating group (3.23 ± 0.27 days) (*P* < 0.05). 3 h, 6 h, and 12 h after the operation, the visual analogue scores (3.82 ± 1.58 points, 2.97 ± 1.53 points, and 1.38 ± 0.57 points) of the patients in the infiltration group were considerably higher than the infiltrating group (2.31 ± 1.46 points, 1.06 ± 1.28 points, and 0.95 ± 0.43 points) (*P* < 0.05). 3 h, 6 h, and 12 h after the operation, the number of patients in the infiltrating group who used tramadol for salvage analgesia (2 cases, 1 case, and 1 case) was notably less than that in the infiltration group (9 cases, 7 cases, and 3 cases) (*P* < 0.05). In short, local anesthetics combined with TAP block can reduce postoperative VAS score and postoperative nausea and vomiting (PONV) score, which also reduced the incidence of postoperative analgesia.

## 1. Introduction

Gynecological laparoscopy has been widely adopted in clinical treatment because of its advantages of small trauma, light pain, and quick recovery [1]. However, due to the different physiques of the patients, the pain is still unbearable. After GLS, patient-controlled intravenous analgesia is commonly adopted, and the analgesic effect is very significant. Due to general anesthesia, it causes more side effects, and it is prone to adverse symptoms such as respiratory depression, nausea, vomiting, and skin itching [2]. Transversus abdominis plane (TAP) block refers to injecting anesthetics into the neurofascial layer between the internal oblique muscle and the transversus abdominis muscle, to block the relevant nerve sensory conduction. Therefore, the pain of the skin, muscles, and peritoneum of the front abdomen is weakened, and a relatively ideal abdominal wall analgesic effect is achieved [3]. In recent years, the application of TAP block in postoperative analgesia has gradually increased. Ping-Chen et al. [4] found that different drug concentrations had a greater impact on laparoscopic surgery, so it was urgent to determine the optimal drug concentration.

With the rapid development of computer image processing technology, its application in medical imaging has been gradually extensive [5]. Ultrasound imaging medicine is one of the important tools for clinicopathological diagnosis, which can improve the efficiency of clinical diagnosis by locating and recognizing ultrasonic images and extracting graphic features. On the premise of feature extraction, image segmentation, image enhancement, and edge features of ultrasonic images, abnormal feature points are extracted from ultrasonic images to enhance the judgment ability of ultrasonic images [6]. Abraham et al. [7] proposed a small porter feature decomposition for the extraction of abnormal feature points in ultrasonic images and decomposed the edge contour features of ultrasonic images. Then, according to the decomposition results, the adaptive information fusion was enhanced to improve the detection of ultrasonic images. Sadek et al. [8] proposed an ultrasonic image localization of correlation characteristics and conducted batch processing of ultrasonic image edges. Based on the above reports, this work proposed an ultrasonic image localization technique based on WTIE algorithm. Firstly, edge feature fusion method was adopted for contour detection of ultrasonic images, color gradient decomposition was carried out in the region, and the ultrasonic image region was fused and filtered. Then, the wavelet transform method was combined to perform feature decomposition and scale template matching on the ultrasound image and process the color feature decomposition value of the ultrasound image, so that the region of the image was equalized. According to the color and texture features of ultrasonic images, the abnormal feature points of the image were located and monitored. Finally, the simulation experiment was utilized for analysis, and the conclusion was reached [9].

In this work, WTIE algorithm was applied to the ultrasound images of 56 patients undergoing GLS. The purpose was to explore the analgesic effect of different concentrations of ropivacaine combined with TAP block on the perioperative period of GLS and provide good clinical adoption reference in the analgesic aspect of GLS.

## 2. Materials and Methods

### 2.1. Selection of Research Subjects

56 patients who were admitted to the hospital from October 17, 2018, to November 19, 2019, that underwent GLS were selected. The average age was 40.32 ± 1.24 years old. All patients were classified as grade I and grade II according to American Society of Anesthesiologists (ASA). The random number table method was utilized to divide the patients into the infiltrating group (*n* = 28) and block group (*n* = 28). The study had been approved by the Medical Ethics Committee of Hospital, and the patients and their families understood the situation of the study and signed the informed consent forms.

Inclusion criteria: (1) patients aged 20–60 years; (2) patients underwent surgery including hysterectomy, ectopic tubal pregnancy removal, and ovarian cyst removal; and (3) patients with clear consciousness and could receive normal examinations.

Exclusion criteria: (1) patients with mental illness; (2) patients with surgery time greater than 3 hours; (3) patients allergic to local anesthetics and drugs during surgery; (4) patients who withdrew from the experiment due to their own reasons; (5) patients with coagulopathy or peptic ulcer.

### 2.2. Observation Indicators

The clinical data of the patients were collected, and various examination indicators of the patient were detected, including blood routine, cardiac color Doppler ultrasound, lung ventilation function, blood biochemical results, infectious disease examinations, electrocardiogram, and chest radiograph. The presurgery inspections were performed in time, to fully understand the diagnosis process. Communications with the attending physician about surgery method and surgery time should be made in time. The patient's mental outlook was observed, to understand the patient's physical condition and take medication. ASA classification: before the anesthesia, the American Society of Anesthesiologists clearly categorized the risk of the upcoming surgery based on the patient's physical condition, which was divided into six levels. VAS score of pain: 0 meant no pain, less than 4 meant slight pain, 5 to 6 indicated moderate pain that can be tolerated, and a score of 7 to 10 indicated severe pain that was unbearable. PONV score: 0 meant no nausea and vomiting, 4 points or less meant slight nausea and vomiting, a score of 5 to 6 indicated moderate nausea and vomiting, and a score of 7 to 10 indicated severe nausea and vomiting. The patient needed to fast for 4 hours before the surgery.

General information of patients including average age, average height, and average weight of ASA classification was counted. The TAP blocking effect was measured after half an hour using the alcohol method to measure the patient's sensation, and the final data were recorded. The amount of anesthesia used was recorded, especially the amount of propofol used during surgery. The analgesic effect of the patients after surgery was recorded, and the VAS score of pain and PONV score were recorded 3 h, 6 h, and 12 h after the surgery. After the surgery, the number of patients using tramadol was recorded at 3 h, 6 h, and 12 h. Finally, the length of stay of all patients was recorded.

### 2.3. TAP Block Method

For TAP block guided by ultrasonic images, TAP localization should be performed first. Firstly, the ultrasonic probe (5.5∼12 MHz) was placed under the xiphoid process to locate the rectus abdominis and the linea alba, and the probe was rotated to move along the costal margin. In the section position, it could be seen that the TAP was located between the rectus abdominis and the transverse abdominis. If TAP was not observed at the sectionals, it was because the transabdominal muscle terminated at the side of the rectus abdominis in some patients. If the probe was then moved along the costal margin to the position of the semilunar line at the lateral margin of the rectus abdominis, the three layers of the abdominal wall can be clearly identified, which were transverse abdominis, internal oblique, and external oblique from inside to outside, respectively. The probe was continuously moved to the midaxillary line, which was moved up and down between the costal margin and the iliac crest, so that the three bases can be clearly seen. The patient was told to lie on the opposite side, and the probe was moved to the direction of the posterior axillary line. It could be seen that the internal oblique muscle and the transverse abdominis were fused into a layer of fascia, which was called the pectoralis lumbar fascia, and was connected with the outer edge of the quadratus psoas. TAP was located between the transverse abdominis muscle and the internal oblique and was connected with the pectoralis lumbar fascia. A slightly mobile ultrasound probe scanned the ideal position, the area around the puncture site was disinfected with Jill iodine, and the ultrasound probe was wrapped in a sterile protective sleeve. The in-plane technique was adopted, and the nerve blocker was inserted from the medial side to the lateral side. When the puncture needle reached the TAP close to the quadratus psoas, if there was no blood loss during the withdrawal, 0.375% ropivacaine 20 mL would be injected, the ultrasonic image would be utilized to observe the diffusion of local anesthetics, and the step of the nerve blocking needle would be adjusted to continue the injection. 30 minutes after the TAP block, the block plane was detected by alcohol method. If the block scope covered T9∼T12, the block effect was considered to be ideal; but if the block effect was not good, the patient would be withdrawn from the study.

Before surgery, patients in the block group were deflated in the abdominal cavity and sutured four holes. On each of the abdominal wall, a hole was made and injected with 5 mL of 0.375% ropivacaine, a total of 20 mL, for infiltration. The infiltrating group received local anesthetics combined with TAP block method for treatment.

### 2.4. Anesthesia Process and Surgical Method

After the TAP block was over, the patient was anesthetized. Both groups of patients were given intravenous anesthesia, and it was necessary to inject etomidate and sufentanil into the patient's veins. After the muscles were fully relaxed, the patient was put on a ventilator, and the working mode, tidal volume, respiratory rate, and respiratory ratio were determined. During surgery, it was necessary to continue to inject propofol for anesthesia and continue to add atracurium according to the actual surgery. The GLS surgery adopted the laparoscopic four-hole method. The specific positions of the four holes were the upper edge of the umbilical chakra, the right McBurney point, two fingers above the attachment between the left umbilical foramen and the left anterior superior spine of the ilium, and site with no blood vessels in the middle and lower abdomen. After surgery, the patients were transferred to the anesthesia recovery room for postoperative observation, and when they recovered consciousness, they were transferred to the general ward.

### 2.5. WTIE Algorithm

Wavelet transform is based on the frequency localization idea of Fourier transform. It is an analysis method in which the window size is fixed, but the shape, time window, and frequency window can be changed, and the local characteristics of the signal can be characterized in the time domain and frequency domain.

If the function *ϕ*(*s*) has finite energy, then, *ϕ*(*s*) ∈ *M*^2^(*T*). The Fourier transform should be conducted on it, and *ϕ*(*s*) satisfies the following equation:

(1) $$\begin{array}{c} B_{\phi }=\int_{T}\frac{{\left|\phi \left(\alpha \right)\right|}^{2}}{\left|\alpha \right|}d\alpha <\infty . \end{array}$$

In equation (1), *B*_*ϕ*_ represents the coefficient of the wavelet function, and then *ϕ*(*s*) is called the mother wavelet. After it is scaled and translated, the wavelet sequence *ϕ*_*a*,*b*_(*s*) can be obtained, and equation is as follows:

(2) $$\begin{array}{c} \phi_{a,b}\left(s\right)=\frac{1}{\sqrt{\left|u\right|}}\phi \left(\frac{s-v}{u}\right)\;u,v\in T;\;u\neq 0. \end{array}$$

In equation (2), *u* represents the scaling factor, which corresponds to frequency information and *v* represents the translation factor, which corresponds to space-time information. For continuous wavelet transform of function *g*(*s*) ∈ *M*^2^(*T*), the calculation is shown as follows:

(3) $$\begin{array}{c} A_{g}\left(u,v\right)=\frac{1}{\sqrt{\left|u\right|}}\int_{T}g\left(s\right)\phi \left(\frac{t-v}{u}\right)ds. \end{array}$$

In equation (3), *A*_*g*_(*u*, *v*) represents the wavelet coefficient. The wavelet function is reconstructed, and the equation is as follows:

(4) $$\begin{array}{c} g\left(s\right)=\frac{1}{B_{\phi }}\int_{-\infty }^{\infty }\int_{-\infty }^{\infty }\frac{1}{u^{2}}A_{g}\left(u,v\right)\phi \left(\frac{s-u}{v}\right)dudv. \end{array}$$

In equation (4), *g*(*s*) represents the wavelet transform function. Since the continuous wavelet transform function is mainly utilized in theoretical analysis, the continuous wavelet and transform should be discretized in the actual application process. Discretizing the scaling factor *u* and the translation factor *v* as *u*=*u*_0_^*j*^ and *v*=*ku*_0_^*j*^*v*_0_, respectively, the time variable is unchanged, and the discrete wavelet function of the continuous wavelet function is as follows:

(5) $$\begin{array}{c} \phi_{j,k}\left(s\right)=u^{-j/2}\phi \left(\frac{s-ku_{0}^{j}v_{0}}{u_{0}^{j}}\right). \end{array}$$

Therefore, the discretized wavelet coefficient is calculated as follows:

(6) $$\begin{array}{c} B_{i,j}=\int_{-\infty }^{\infty }g\left(s\right)\phi_{j,k}^{\circ }\left(s\right)ds. \end{array}$$

The inverse wavelet transform for discretization is as follows:

(7) $$\begin{array}{c} g\left(s\right)=b\sum_{j=-\infty }^{\infty }\sum_{k=-\infty }^{\infty }b_{j,k}\phi_{j,k}\left(s\right). \end{array}$$

In equation (7), *b* is a constant. It can be seen that the smaller the *u*_0_ and *v*_0_, the higher the signal reconstruction accuracy.

Infrared image is a two-dimensional discrete image *A*(*u*, *v*), which can be regarded as a two-dimensional matrix and subjected to two-dimensional wavelet transformation. Then, it is decomposed into low-frequency components PP1, PQ1, QP1, and QQ1 at each resolution of each layer, and high-frequency components PP2, PQ2, QP2, and QQ2 in the three directions of horizontal, vertical, and diagonal. The schematic diagram of wavelet transform is shown in Figure 1, and the image reconstruction process is just the opposite.

A threshold function is adopted to modify the positive wavelet coefficients. Commonly utilized threshold functions include hard threshold functions and soft threshold functions. It is assumed that *A* is a wavelet function, and *A*_*S*_ is threshold-treated wavelet coefficient, where *S* is the threshold. The hard threshold function means that when the absolute value of the wavelet coefficient is less than the threshold, it is equal to 0, and when it is greater than or equal to the threshold, it remains unchanged. The equation is as follows:

(8) $$\begin{array}{c} A_{s}=\left\{\begin{array}{cc} A, & \left|A\right|\geq S\\ 0, & \left|A\right|<S \end{array}\right). \end{array}$$

The hard threshold function means that when the absolute value of the wavelet function is less than the threshold, it is equal to 0, and when it is greater than or equal to the threshold, the threshold is subtracted. The equation is as follows:

(9) A=ssignAA−SA≥S0A<S.

The key point of threshold denoising is the choice of threshold. If the choice of threshold is too large, it is possible to delete a lot of important information, and if the threshold is too small, it may affect the denoising effect. The VisuShrink threshold and the universal unified threshold is adopted. The calculation equation of the threshold *S* is as follows:

(10) $$\begin{array}{c} S=\sigma_{m}\sqrt{2\;\ln\;M}. \end{array}$$

In equation (10), *σ*_*m*_ represents the standard deviation of noise and *M* represents the length of the signal. Moreover, for the details of high-frequency components, the adoption of coefficient transformation can improve the contrast of the image and enhance the visual effect. The equation is as follows:

(11) $$\begin{array}{c} S_{\text{OUT}}=H\left(S_{A}+f\right). \end{array}$$

In equation (11), *S*_OUT_ represents the wavelet function after detail enhancement, *S*_*A*_ represents the wavelet function after threshold processing, *H* represents the gain factor, and *f* represents the offset.

### 2.6. Statistical Methods

Data processing adopted SPSS19.0 version statistical software analysis, measurement data conformed to normal distribution were recorded in the form of mean ± standard deviation $\left(\bar{x}\pm s\right)$, and count data were recorded as percentage (%). The surgery time, length of stay, dosage, pain VAS score, and PONV scores of two groups were all analyzed by variance. The difference was considerable at *P* < 0.05.

## 3. Results

### 3.1. Statistics of General Information of Patients

There was no considerable difference in the average age, average weight, average height, and ASA classification results between the two groups (*P* > 0.05) (Figure 2). The GLS surgery received by the two groups of patients included ovarian cyst removal, hysteromyoma removal, and subtotal hysterectomy. Among them, of the majority of patients undergoing ovarian cyst removal, no notable difference was shown within or between groups (*P* > 0.05) (Figure 3).

### 3.2. Ultrasound Image of Gynecological Abdominal Cavity during Perioperative Period

There was a huge cystic mass in the peritoneal cavity of the ovarian cyst, with multiple compartments and compartments inside, large intra-atrial sound transmission difference, and dense spot echo. Other parts showed multiple vesicle-like aggregation. Ultrasonography showed a large amount of effusion in the abdominal cavity, with poor sound transmission, which was manifested as dense punctate echo. Original abdominal mass and whole volume manifestation were confined to the lower abdomen and pelvic cavity (Figure 4).

Uterine fibroids showed that the original lesion still had an echo mass with a diameter similar to that of the original lesion. This was the result of inflammatory response edema in local tissues after lesion coagulation. When ultrasound imaging was adopted for inspection, it can be seen that the original lesion still had echogenic light mass, and the diameter of the echogenic light group was generally significantly smaller than that of the original lesion, with irregular boundary and blood vessels piercing into it. This was the result of solidification of a fibroid or adenomyoma into scar tissue, which was a normal phenomenon (Figure 5).

### 3.3. Distribution of Blocking Planes

The anterior abdominal skin, muscles, and parietal peritoneum were innervated by T9∼L1 anterior spinal nerves. After these spinal nerves left the intervertebral foramen, the anterior branch passed through the lateral abdominal wall muscles and run along the transverse abdominal muscle plane to innervate the anterior abdominal muscles and skin. The T9∼T12 anterior branch entered the TAP layer from the inside of the anterior axillary line. Local anesthetics combined with TAP block were received by the two groups of patients, and no considerable difference in the block distribution was found after half an hour of surgery, as shown in Figure 6(*P* > 0.05), and the block effect of the two groups was ideal.

### 3.4. Propofol Dosage during Surgery

The dosage of propofol in the block group (313.23 ± 19.67 mg) was substantially lower than that of the infiltration group (377.67 ± 21.56 mg) (*P* < 0.05) (Figure 7). In terms of surgery time, no evident differences between the two groups were found (*P* > 0.05) (Figure 8). The hospitalization time of patients in the block group (2.14 ± 0.18 days) was significantly shorter relative to the infiltrating group (3.23 ± 0.27 days) (*P* < 0.05) (Figure 9).

### 3.5. VAS Score and PONV Score for Postoperative Pain

3 h, 6 h, and 12 h after the operation, the VAS scores (3.82 ± 1.58 points, 2.97 ± 1.53 points, and 1.38 ± 0.57 points) of the infiltrating group were greatly superior to the block group (2.31 ± 1.46 points, 1.06 ± 1.28 points, and 0.95 ± 0.43 points) (*P* < 0.05) (Figure 10); PONV score of the infiltrating group (1.84 ± 0.65, 1.53 ± 0.82, and 1.16 ± 0.36) was notably less than the block group (2.37 ± 0.46, 1.94 ± 0.52, and 1.57 ± 0.42) (*P* < 0.05) (Figure 11).

### 3.6. Tramadol Used for Postoperative Salvage Analgesia

3 hours after the operation, 2 patients in the block group used tramadol for salvage analgesia. 6 hours after the operation, 1 patient in the block group used tramadol. 12 hours after the operation, one patient in the block group was treated with tramadol. 3 hours after the operation, 9 patients in the infiltration group used tramadol. 6 hours after the operation, 7 patients in the infiltration group used tramadol. 12 hours after the operation, 3 patients in the infiltration group received tramadol. The difference between the two groups at each time point was obvious (*P* < 0.05) (Figure 12).

## 4. Discussion

Pain after laparoscopic gynecological surgery includes pain at the incision site of abdominal surgery, pain in internal organs around organs, pain caused by phrenic nerve stimulation, and pain caused by tissue inflammation caused by surgery. Blanco et al. [10] deemed that the utilization of posterior approach for TAP block had a certain relief effect on peripheral visceral pain. Öksüz et al. [11] pointed out that the TAP block method can reduce the pain in the front of the abdomen, but it cannot reduce the pain in the internal organs. Studies have reported that intravenous injection of propofol before surgery can prevent the synthesis of cyclooxygenase and reduce the prostatic hormone content of the surgical site, thereby achieving the purpose of analgesia [12]. This work revealed that when patients received propofol combined with TAP block, in contrast to the infiltrating group, the dose of propofol used in the block group was greatly reduced during surgery, which can significantly reduce the pain VAS score after surgery, and the results were consistent with the above research results.

Previous studies have pointed out that local anesthetics combined with nerve block can reduce the dosage of opioid analgesics [13]. The results showed that the VAS scores and PONV scores of patients with TAP block decreased evidently at 3 h, 6 h, and 12 h after surgery, and the number of patients who used tramadol for analgesic remedy after surgery was reduced, which greatly improved patient satisfaction. The results were consistent with those of Zhang et al. [14].

TAP block adopted the water separation method to separate and diffuse local anesthetics and utilized local anesthetics to infiltrate the blocked nerves. The low concentration of local anesthetics will make the analgesic effect insignificant, while the high concentration will increase the drug concentration in plasma. Therefore, TAP block requires the adoption of appropriate drug concentration and dosage [14]. In this work, 20 mL of 0.375% ropivacaine was used to observe the block plane distribution between the two groups within 30 minutes after the TAP block, and the difference was not considerable (*P* < 0.05). Sun et al. [15] performed GLS on women after TAP block, and the concentrations of ropivacaine were 0.25%, 0.40%, and 0.45%, respectively, and the dosage was 40 mL. Plasma levels of ropivacaine in each group were measured after TAP block. The results showed that the maximum blood concentration changed with the injection. Adverse reactions to local anesthetics generally occurred within 10 minutes after completion of TAP block. The results of this work were different from those of the above studies, which may be related to the cases of the patients in this work, and it should further determine the concentration of ropivacaine in the blood.

## 5. Conclusion

Wavelet transform was adopted to enhance the ultrasound images, and it was revealed that the algorithm can enhance the image contrast, and the denoising effect was very strong. Ultrasound imaging technology was utilized to intuitively guide the direction of needle insertion during puncture, and it was proved that 0.375% ropivacaine can accurately enter the TAP, maximizing the analgesic effect. It also reduced the VAS score and PONV score of patients after surgery and reduced the incidence of postoperative analgesia. Moreover, the amounts of opioid analgesics during the GLS perioperative period and the occurrence of malignant reactions were also reduced. In contrast to the previous intravenous analgesia treatment, it greatly improved the comfort and satisfaction of patients after surgery. The limitation of this study is that only the clinical effects of the two groups of patients were compared, yet the concentration of ropivacaine in the blood was not further measured. In conclusion, local anesthetic combined with TAP block was used in this work, which provided a good reference for clinical GLS perioperative period.

## Figures and Tables

**Figure 1:** Schematic diagram of two-dimensional wavelet transform.

**Figure 2:** Contrast of general conditions of the two groups of patients.

**Figure 3:** The proportion of ovarian cyst removal, hysteromyoma removal, and subtotal hysterectomy.

**Figure 4:** Ultrasound image of ovarian cyst of a female patient who underwent GLS (38 years old).

**Figure 5:** Ultrasound image of uterine fibroids of a female patient who underwent GLS (35 years old).

**Figure 6:** Contrast of block plane distribution.

**Figure 7:** Contrast of propofol dosage during surgery between the two groups. Note: ^*∗*^ meant *P* < 0.05 versus infiltrating group, the same for Figures 8 and 9.

**Figure 8:** Contrast of surgery time between two groups of patients.

**Figure 9:** Contrast of length of stay between two groups of patients.

**Figure 10:** VAS score of postoperative pain of patients. Note:^*∗*^ meant *P* < 0.05 versus infiltrating group.

**Figure 11:** PONV score of postoperative pain of patients. Note:^*∗*^ meant *P* < 0.05 versus infiltrating group.

**Figure 12:** Contrast of the number of cases using tramadol in the two groups. Note: ^*∗*^ meant *P* < 0.05 versus infiltrating group.

## Data Availability

No data were used to support this study.
